# miR-188-3p abolishes germacrone-mediated podocyte protection in a mouse model of diabetic nephropathy in type I diabetes through triggering mitochondrial injury

This article has been retracted.

**DOI:** 10.1080/21655979.2021.2012919

**Published:** 2022-01-05

**Authors:** Yunguang Wang, Fangfang Feng, Wenfang He, Lifang Sun, Qiang He, Juan Jin

**Affiliations:** a Department of Critical Care Medicine, Affiliated Hangzhou First People’s Hospital, Zhejiang University School of Medicine, Hangzhou, P. R. China; b Department of Nephrology, Zhejiang Provincial People’s Hospital, Affiliated People’s Hospital, Hangzhou Medical College, Hangzhou, P.R China; c Department of Tuberculosis, Hangzhou Red Cross Hospital, Hangzhou, P.R China; d Department of Tuberculosis, Affiliated Hangzhou Chest Hospital, Zhejiang University School of Medicine, Hangzhou, P.R China

**Keywords:** Diabetic nephropathy, podocyte, germacrone, miR-188-3p, mitochondrial damage

## Abstract

Mitochondrial injury-triggered podocyte apoptosis is a major risk factor for diabetic nephropathy (DN). However, the detailed relationship between mitochondrial homeostasis and podocyte apoptosis remains unclear. The present study aimed to explore the role and functional mechanism of germacrone in DN in type I diabetes (type I DN). A mouse model of type I DN was established by injecting streptozocin, and a podocyte injury model was constructed using high glucose (HG) induction. Histopathology was detected by hematoxylin and eosin and periodic acid-Schiff staining. Transmission electron microscopy and flow cytometry were used to evaluate the mitochondrial function. Germacrone simultaneously reduced blood glucose, 24 h proteinuria, and other nephrotic symptoms in a type 1 DN mouse model. Moreover, germacrone protected against mitochondrial damage, limited reactive oxygen species (ROS) accumulation, and restored glutathione peroxidase (GPX) activity and GPX4 protein expression, subsequently preventing podocyte apoptosis. Mechanistically, the increased miR-188-3p expression in type I DN mice was reversed in germacrone-challenged DN mice. HG induced miR-188-3p expression and the miR-188-3p antagonist abolished the HG-mediated increase in ROS. Notably, miR-188-3p was found to have a therapeutic effect against DN by aggravating mitochondrial damage and podocyte apoptosis. Germacrone alleviates DN progression in type I diabetes by limiting podocyte apoptosis, which was partly counteracted by miR-188-3p upregulation. The combination of germacrone and miR-188-3p antagonists is expected to be an effective therapeutic strategy for DN.

**Abbreviations DN:** diabetic nephropathy; Type I DN: DN in Type I diabetes; STZ: streptozocin; ROS: reactive oxygen species; NcRNAs: non-coding RNAs; UTR: untranslated regions; NC: negative control; BUN: blood urea nitrogen; BUA: blood uric acid; Ucr: urine creatinine; Scr: serum creatinine; PAS: Periodic Acid-Schiff; IF: Immunofluorescence; FISH: Fluorescence in situ hybridization; TUG1: taurine upregulated gene 1; GPX: Glutathione Peroxidase; GPX4: glutathione peroxidase 4; EMT: epithelial-mesenchymal transition

## Introduction

Diabetic nephropathy (DN) is the predominant cause of end-stage renal disease (ESRD) worldwide [1] and is also the leading cause of mortality in type 1 diabetes patients [2]. The hallmark features of DN include an increased amount of albuminuria, accompanied by swelling of the glomerular basement membrane and mesangial nodular hyperplasia [3,4]. Microalbuminuria, as the earliest clinical phenotype of DN, has a cumulative lifetime incidence of approximately 50% in type 1 diabetes, and increases at a rate of approximately 2%–3% annually [5]. Notably, 25% of type 1 diabetes patients with DN progress to ESRD [6]. Therefore, there is a considerable challenge in preventing DN in type I diabetes patients.

The development of DN is frequently characterized by morphological and pathological changes in podocytes, including podocyte hypertrophy, apoptosis, detachment, and epithelial-mesenchymal trans-differentiation [7–9]. Podocytes, which are highly differentiated glomerular epithelial cells, are crucial for maintaining the glomerular filtration barrier [8,10]. Glomerular filtration function is an imperative evaluator of urinary protein and chronic kidney disease, and podocytes play a leading role in this process [11,12]. Podocyte apoptosis is closely related to mitochondrial injury in DN [13,14]. Accumulating evidence has shown that reactive oxygen species (ROS) can trigger cell apoptosis in the process of type I and II diabetes with DN [15–17]. Hyperglycemia-induced mitochondrial injury leads to the abundant accumulation of ROS, subsequently triggering oxidative stress, which is considered a critical contributor to podocyte apoptosis and loss in DN [13,14]. Accumulating studies have shown that mitochondrial injury-mediated podocyte apoptosis and loss are tightly correlated with DN progression in type I diabetes, however, the underlying mechanism remains unclear and requires further investigation.

Rhizoma curcuma is a common traditional Chinese medicine with anti-inflammatory and antioxidant effects [18]. Germacrone, the major bioactive constituent of Rhizoma curcuma, is widely known as an antibacterial, antifungal, antitumor, antioxidant, and anti-tussive agent [19,20]. Germacrone mediates cell cycle arrest and the mitochondrial injury pathway in various cancers [21,22]. Germacrone plays a neuroprotective role by protecting against oxygen-glucose deprivation/reperfusion injury [23]. Germacrone reduces cisplatin-induced nephrotoxicity by inhibiting organic cation transporters [24]. Substantial evidence has shown that germacrone has strong antioxidant and anti-apoptotic effects, however, the role of germacrone in the development of DN remains unclear.

Currently, researchers have noticed that the participation of non-coding RNAs (ncRNAs) in DN development, and the mechanisms of different types of ncRNAs have also been clearly clarified [25–27]. miRNAs are common ncRNAs with small nucleic acids that can bind to the 3ʹ-untranslated regions of their target mRNAs [28]. Microarray analysis suggests that miRNAs are involved in the course of DN, and miRNAs play multiple roles in the pathogenesis of DN, including inflammation, apoptosis, autophagy, and cell proliferation [29,30]. miR-188-3p sponged the tumor necrosis factor receptor-associated factor 3 pathway to prevent cell apoptosis, contributing to the treatment of ischemia/reperfusion injury [31]. miR-188-3p inhibition contributes to the promotion of apoptosis in spermatogenic cells [32]. Although accumulating evidence has indicated that miR-188-3p exerts anti-apoptotic effects in several cell types, its function in podocyte apoptosis and DN progression remains unclear.

In the present study, we attempted to illustrate the role and functional mechanism of germacrone in type I DN. Additionally, we aimed to explore the role of miR-188-3p in germacrone-challenged DN mice. Our findings provide novel insights into the management of type I DN.

## Materials and methods

### Animals and treatments

Eighty male C57BL/6 J mice (8-weeks old) were obtained from the China Three Gorges University (Yichang, China). The mice were intraperitoneally administered streptozocin (STZ) at 40 mg/kg/day (S0130, Sigma-Aldrich, MO, USA) for five consecutive days to establish a type I diabetic mouse model [33]. The blood glucose of mice > 16.7 mmol/L was considered as hyperglycemic. The diabetic mice were divided into two groups (n = 6/each of group): model (C57BL/6 J+ STZ) and experimental (C57BL/6 J+ STZ+Germacrone). The experimental group was treated with germacrone (2 mg/kg/day). For the inhibitor assay, the mice with type I diabetes were divided into four groups: model group (C57BL/6 J+ STZ), experimental group 1 (C57BL/6 J+ STZ+germacrone), experimental group 2 (C57BL/6 J+ STZ+germacrone+miR-188-3p agomir), and experimental group 3 (C57BL/6 J+ STZ+germacrone+agomir negative control [NC]). For injection of miRNAs, each mouse was injected with 10 nmol miR-188-3p agomir or 10 nmol NC into the tail vein every three days. The agomirs were diluted with Entranster *in vivo* transfection reagent (Engreen, Beijing, China). All animal experiments were performed in compliance with the guidelines of Zhejiang Provincial People’s Hospital and were approved by the local institution and ethics committee of Zhejiang Provincial People’s Hospital (20210180).

### Podocyte culture

Primary mouse podocytes, MPC5, were acquired from the Institute of Basic Medicine, Chinese Academy of Medical Sciences. Podocytes were cultured in RPMI-1640 medium (SH30809.01B, HyClone, UT, USA) supplemented with 10% FBS and 100 U/mL penicillin-streptomycin (DY14011, HyClone) at 37°C. Subsequently, the cells were cultured overnight at 37°C for 10–12 days in serum-free medium. Podocyte differentiation was induced with 25.5 mM mannitol or 25.5 mM glucose.

### Quantification of BUN, BUA, Ucr and Scr

The fasting blood glucose level was monitored every 4 weeks using an Omron Glucometer (HEA-230, Kyoto, Japan), and 24 h urine was collected at 2-week intervals and stored at − 80°C until analysis. At the end of the study, blood samples were collected from the retro-orbital plexus. Kidney tissues were harvested for histological assessment and total protein or RNA extraction. Urine proteinuria, blood urea nitrogen (BUN), and blood uric acid (BUA) levels were analyzed using a fully automatic biochemical analyzer (7020, Hitachi, Tokyo, Japan), and urine creatinine (Ucr; EY3923, E-research BioTech, Shanghai, China) and serum creatinine (Scr; LE-M1588, Lai-er BioTech, Hefei, China) were measured using the homologous ELISA kits.

### Histological staining

The kidneys were fixed in 4% PFA (30,525–89-4, Sinopharm, Shanghai, China), dehydrated, and embedded in paraffin. The paraffin-embedded tissues were cut into sections of 5 μm thickness. The sections were dewaxed and subjected to hematoxylin (CTS-1099, MXBio, Fuzhou, China) and 0.5% eosin (71,014,544, Sinopharm). Subsequently, slices were mounted with neutral gum (G8590; MAIRUI, Shanghai, China). Images of glomerular and mesangial membrane morphologies were observed under a microscope.

### Periodic acid-Schiff (PAS) staining

Renal tissue sections were dehydrated, and 5 μm paraffin-embedded sections were stained with 10 g/L periodic acid solution (10,450–60-9, Nanjing Reagent, Nanjing, Chin) for 15 min. Next, the slices were incubated with Schiff dye solution (DG0005, Leagene Biotech, Beijing, China) for 1 h at 37°C, stained with hematoxylin (CTS-1099, MXBio) for 5 min, and mounted with coverslips.

### Immunofluorescence staining

The treated cells were fixed with 4% PFA for 10 min and permeabilized with 0.1% Triton X-100 (ST795, Beyotime Biotechnology, Jiangsu, China) for 5 min. The slices were blocked in 5% BSA at 25°C for 1 h, and subsequently incubated with primary antibodies against podocin (ab50339, Abcam, Cambridge, UK, 1:200) and nephrin (ABIN2177857, antibodies-online.com, Aachen, Germany, 1:200), and synaptopodin (ab224491, Abcam, 1:100) at 4°C overnight. The following day, sections were stained with horseradish peroxidase (HRP)-conjugated secondary antibody goat anti-rabbit IgG (BA1032, Boster Biological Technology, Wuhan, China), and the cell nucleus was stained by DAPI (C1002, Beyotime Biotechnology).

### Fluorescence in situ hybridization (FISH)

To evaluate miR-188-3p expression in STZ-induced DN mice, a FISH assay was performed using a Cy3-labeled miR-188-3p probe. The miR-188-3p probe (5ʹ-DIG- TGCAAACCCTGCATGTGGGAG-DIG-3ʹ) was designed and synthesized by Abace Biotechnology (Beijing, China). The miR-188-3p signals were detected with a FISH Tag™ kit (Abace Biotechnology) according to the manufacturer’s instructions. The specimens were visualized using an inverted fluorescence microscope (BX53; Olympus, Japan).

### RNA isolation and real-time PCR

Total RNA was extracted from kidney samples using TRIzol reagent (15596–026; Ambion, TX, USA) according to the manufacturer’s instructions. The RNA was reverse transcribed into cDNA using a reverse transcription kit (AT101-02; TransGen Biotech, Beijing, China). The primer sequences of mmu-miR-188-3p were as follows: forward, 5ʹ-TGCGCCTCCCACATGCAGGGT-3ʹ; loop: 5ʹ-GTCGTAGGATAGTGCAGGCAAACGAGGTATTACT-3ʹ, reverse: 5ʹ-CCAGTGCAGGGTCCGAGGTAT-3ʹ. Next, miR-188-3p expression was amplified by SYBR Green Master Mix (Q111-02; Vazyme, Jiangsu, China) according to the manufacturer’s data sheets, and calculated by the comparative Ct method and normalized to the housekeeping gene U6 (U6-Forward, 5ʹ-CGCTTCGGCAGCACATATAC-3; U6-Reverse, 5ʹAAATATGGAACGCTTCACGA-3ʹ); The primers were designed by using Primer Premier 5 software (Premier Biosoft International, CA, USA).

### Detection of ROS level

ROS levels were evaluated using the DCFH-DA ROS Assay kit (S0033; Beyotime). Briefly, kidney tissue homogenates were incubated with 10 μmol/L DCFH-DA for 30 min at 37°C in the dark. The fluorescence intensity was monitored at a wavelength of 485 nm using a fluorescence spectrophotometer (PerkinElmer, MA, USA). To detect intracellular ROS levels, the ROS-sensitive probe H2DCFDA (HY-D0940; MedChemExpress, NJ, USA) was used. MPC5 podocytes were incubated with 5 μM staining solution in PBS for 30 min in the dark at 37°C, then harvested with 0.05% trypsin-EDTA solution, suspended in fresh medium, and immediately analyzed with a flow cytometer.

### Glutathione peroxidase (GPX) activity

We digested and centrifuged 8%–10% kidney tissues to collect the supernatants. GPX activity was assessed using the Glutathione Peroxidase Cellular Activity Assay Kit (CGP-1, Sigma-Aldrich) in the supernatants. Briefly, 50 μL kidney tissue homogenates were co-incubated with 890 μL GPx assay buffer, 50 μL NADPH Assay Reagent, and 10 μL t-Bu-OOH (30 mM) for 30 min at 37°C, and the results were monitored at a wavelength of 340 nm using a spectrophotometer (PerkinElmer).

### Transmission electron microscopy (TEM)

Fresh kidney tissues were fixed in fixative for 6 h and continuously fixed in 0.1 M phosphate buffer (1% osmic acid) for 2 h. After washing three times with 0.1 M phosphate buffer, the tissues were dehydrated and embedded in Epon-812 (S2659, XinwangWeiTuo Technology, Peking, China). The paraffin-embedded tissue was cut into sections of 60–80 nm in thickness. The sections were then dehydrated and stained using uranyl acetate-lead citrate, and images were observed using a transmission electron microscope (HT7700, Hitachi).

### Western blot

Total protein was extracted with RIPA buffer (P0013B, Beyotime) mixed with a protease inhibitor cocktail (G1205, Servicebio, Wuhan, China). The protein bands were incubated with primary antibodies against GAPDH (Ab181602, Abcam, 1:1000), GPX4 (Ab125066, Abcam, 1:3000), Prodocin (Ab50399, Abcam, 1:1000), and nephrin (Ab58968, Abcam, 1:1000) overnight at 4°C. HRP-conjugated goat anti-rabbit or anti-mouse IgG (BA1054, BA1053, BOSTER, Wuhan, China, 1:5000) was used as the secondary antibody for 1 h at 25°C. The blots were visualized using the ECL chemiluminescence reagent kit (Millipore, MA, USA) and photographed on a ChemiDoc™ MP Imaging System (Bio-Rad, CA, USA).

## Statistical analysis

All measurements were performed in at least three independent experiments. The data are expressed as the mean ± SEM. SPSS 25.0 software was used for statistical analysis. Differences among groups were analyzed using a two-way ANOVA or two-tailed Student’s t-test. Statistical significance was set at p < 0.05.

## Results

In this study, we revealed that germacrone protected against mitochondrial malfunction and podocyte apoptosis in a mouse model of DN with type I diabetes. Mechanistically, miR-188-3p dramatically counteracted the effects of germacrone, triggering oxidative stress and subsequently inducing podocyte apoptosis. Our findings may provide innovative ideas for the treatment of DN in type I diabetes.

## Germacrone relieves the development of type I DN

The STZ-injected C57BL/6 J mice developed type I diabetes at 9 weeks, when the blood glucose surpassed 16.7 mmol/L after continuous STZ treatment (Figure 1(a)). Renal function was monitored for each group. BUN, Scr, BUA, and 24 h proteinuria were robustly increased in the STZ-injected C57BL/6 J mice, while Ucr displayed a declining tendency (Figure 1(b–f)). These characteristics were reversed by germacrone treatment (2 mg/kg/day), as the blood glucose and kidney function indicators dramatically decreased and returned to normal levels (Figure 1(b–f)). Histological examination revealed glomerular hypertrophy and mesangial matrix expansion to fluid vacuoles in STZ-injected mice (Figure 1(g–h)), which apparently indicated symptoms of DN. Germacrone treatment markedly ameliorated glomerular hypertrophy and recovered the normal mesangial membrane (Figure 1(g–h)). These findings suggest that germacrone may relieve the development of DN.

**Figure 1.** Effects of germacrone on type I diabetic nephropathy (DN) symptoms. (a) Blood samples were collected from wild-type (WT), streptozocin (STZ)-induced mice. BG was determined using an Omron Glucometer, **P < 0.01. (b–f) Urine and blood samples of WT, STZ-induced mice and STZ+germacrone co-treated mice were collected. Subsequently, 24 h proteinuria, BUN, and BUA were analyzed using a fully automatic biochemical analyzer, and Ucr and Scr were measured with the homologous ELISA kits, **P < 0.01. (g–h) Kidney tissues obtained from the different groups were cut into paraffin sections. Then, the sections were stained by hematoxylin and eosin (HE) and PAS. Scale bar: 100 μm. Magnification: ×400, **P < 0.01. BG: blood glucose, Pro: proteinuria, BUN: blood urea nitrogen, Scr: serum creatinine, Ucr: urine creatinine, BUA: blood uric acid, Ger: Germacrone.

## Germacrone protects against podocyte apoptosis via preventing mitochondrial damage in STZ-induced diabetic mice

Podocytes, also called glomerular epithelial cells, are specially differentiated cells in the glomerulus, which is a critical element for maintaining glomerular filtration function [34]. Podocyte disruption and apoptosis have been shown to induce unfavorable reactions in DN progression. Oxidative stress caused by mitochondrial damage is the center of podocyte apoptosis [33]. We found that the morphology of the mitochondria was severely deteriorated in the STZ-induced diabetic mice, the membrane and cristae were broken, and the structure was completely out of shape (Figure 2(a)). There was an increased accumulation of ROS and reduction of GPX, which were rescued by germacrone treatment (Figure 2(b–c)). Western blotting also showed that germacrone elevated the expression of recombinant glutathione peroxidase 4 (GPX4), which is a pivotal enzyme regulated by glutathione (GSH) and decreased in DN mice (Figure 2(d)). Mitochondrial damage induces podocyte apoptosis under pathological conditions. Protein expression and distribution of podocin and nephrin, which are biomarkers of podocytes, were monitored. The diminished expression of podocin and nephrin in STZ-induced DN mice and high glucose-induced MPC5 podocyte cells were observed (Figure 2(d) & Fig. S1), indicating that mitochondrial damage may induce podocyte apoptosis. Interestingly, germacrone reversed this result and prevented podocyte apoptosis (Figure 2(d) & Fig. S1). In general, our findings suggest that germacrone may resist podocyte apoptosis by repairing mitochondrial function.

**Figure 2.** Role of germacrone on podocyte apoptosis in STZ-induced DN mice. (a) Kidney sections in WT, STZ-induced mice and STZ+germacrone co-treated mice were magnified by electron microscopy, the red arrows point to the damaged mitochondria, magnification: ×7000, scale bar: 1 μm. (b) Mitochondrial reactive oxygen species (ROS) production was evaluated in the above groups with a DCFH-DA ROS Assay kit, **P < 0.01. (c) Measurement of GPX activity was assessed with Glutathione Peroxidase Cellular Activity Assay Kit, **P < 0.01. (d) The expressions of GPX4, podocin, and nephrin proteins were detected by Western blots in each group, with GAPDH serving as a loading control. (e) Quantitative analysis of protein expression including GPX4, podocin, and nephrin. **P < 0.01.

## miR-188-3p is involved in the germacrone-mediated improvement of DN

miR-188-3p can combine with other ncRNAs and exert multiple effects in the majority of cell types. In the present study, increased miR-188-3p expression was observed in STZ-challenged DN mice compared to that in healthy subjects by FISH assay (Figure 3(a)). Moreover, real-time PCR experiments also revealed that miR-188-3p expression in STZ-induced podocytes was higher (Figure 3(b)). Conversely, treatment with germacrone reduced miR-188-3p expression (Figure 3(a–b)). Thus, we speculated that miR-188-3p may be involved in the germacrone-mediated improvement of DN.

**Figure 3.** miR-188-3p is involved in the progression of DN. (a) FISH assay was performed to value the distribution of miR-188-3p in WT, STZ-induced mice and STZ+germacrone co-treated mice. Magnification: ×400. Scale bar: 100 μm. (b) Real-time quantitative PCR was used to detect the RNA level of miR-188-3p *in vivo*, with U6 serving as the internal control, **P < 0.01.

## miR-188-3p expands the ROS oxidation products in HG-induced podocytes

To ascertain the mechanism of miR-188-3p in the field of MPC5, podocytes were used to explore its function *in vitro*. First, we confirmed that miR-188-3p agomir/antagomir worked in MPC5 cells (Figure 4(a)). Subsequently, miR-188-3p antagomir (UGCAAACCCUGCTUGUGGGTG) was transfected into mannitol and HG-treated cells. Consistent with the *in vivo* results, the content of miR-188-3p was extremely high in HG-induced podocytes, and miR-188-3p antagomir exposure significantly abolished the promotion effects of HG (Figure 4(b)). Additionally, the production of ROS was elevated in HG-induced podocytes, which was rescued by the addition of miR-188-3p antagomir (Figure 4(c-d)). It is evident that miR-188-3p induces the production of excessive ROS in HG-exposed cells, which may be the fundamental event of podocyte apoptosis in DN.

**Figure 4.** The role of miR-188-3p on the ROS in high glucose-induced podocytes. (a) The miR-188-3p agomir/antagomir were transfected in mouse podocytes MPC5 cells to confirm the efficiency using RT-qPCR, **P < 0.01. (b) The RNA levels of miR-188-3p were detected in mannitol, glucose, miR-188-3p antagomir, and vehicle stimulated podocytes, **P < 0.01. (c–d) DCFH-DA ROS Assay kit was used to detect the production of ROS in different condition-induced podocytes.

## miR-188-3p agomir prevents the effect of germacrone on DN

Subsequently, we used miR-188-3p agomir to intervene in STZ-induced C57BL/6 J mice, recognizing the role of miR-188-3p in type I DN mice. With the forceful intervention of miR-188-3p agomir, renal analysis indicators, including proteinuria, BUN, Scr, BUA, and Ucr were completely dysregulated, even in the presence of germacrone treatment. The improvement in 24 h proteinuria, BUN, Scr, BUA, and Ucr caused by germacrone were reversed by the challenge of miR-188-3p agomir (Figure 5(a–f)). Hematoxylin and eosin and PAS staining indicated that kidney tissue showed glomerular hypertrophy, the vacuole became plump, and the membrane thickened in the presence of miR-188-3p agomir and germacrone compared to that in germacrone alone-challenged mice (Figure 5(g–h)). Taken together, these results further verify that the miR-188-3p agomir can forestall the positive impact of germacrone on DN.

**Figure 5.** Role of miR-188-3p on the therapeutic effect of germacrone on DN. (a) Blood samples were collected from WT, STZ-induced mice and blood glucose was determined using an Omron Glucometer, **P < 0.01. (b–f) Urine and blood samples of WT, STZ-induced mice, STZ+germacrone co-treated mice, STZ+germacrone+miR-188-3p agomir co-induced mice and STZ+germacrone+miR-188-3p agomir NC co-treated mice were collected, and 24 h proteinuria, BUN, and BUA were analyzed using a Fully automatic biochemical analyzer. Ucr and Scr were measured with the homologous ELISA kits, **P < 0.01. (g–h) Kidney paraffin sections obtained from the different groups underwent HE and PAS staining. Magnification: ×400. Scale bar: 100 μm.

## miR-188-3p blocks the function of germacrone via promoting the number of podocytes

Next, the underlying mechanism of miR-188-3p in DN was explored. TEM analysis indicated that germacrone-mediated improvement in mitochondrial damage was reversed by miR-188-3p agomir, showing mitochondrial swelling, vacuole formation, and mitochondrial cristae tattered in kidney tissues (Figure 6(a)). Additionally, ROS production was reduced in germacrone-challenged DN mice, whereas miR-188-3p agomir treatment restored ROS levels to a high level (Figure 6(b)). Excessive miR-188-3p was observed in type I DN mice as before, and miR-188-3p agomir notably elevated its expression compared to that in the germacrone-challenged group (Figure 6(c)). Similar to the tendency of miR-188-3p expression in the STZ-induced DN mice, a significant reduction in the GPX4, podocin, and nephrin proteins was detected in DN mice, and miR-188-3p agomir also prevented the promotion role of germacrone on their expression (Figure 6(d)). These data confirm that miR-188-3p inhibits mitochondrial oxidation function, and restores the number of podocytes.

**Figure 6.** The blocking role of miR-188-3p on the function of germacrone by mediating podocyte apoptosis. (a) Micrographs of kidney sections in WT, STZ-induced mice, STZ+germacrone co-treated mice, STZ+germacrone+miR-188-3p agomir co-induced mice and STZ+germacrone+miR-188-3p agomir NC co-treated mice were recorded by electron microscopy; the red arrows point to the damaged mitochondria. Scale bar: 1 μm. Magnification: ×7000. (b) Mitochondrial ROS production was evaluated in the above groups with a DCFH-DA ROS Assay kit, **P < 0.01. (c)-(d) RNA level of miR-188-3p and GPX4, podocin, and nephrin proteins were measured in different groups, **P < 0.01. (e) Quantitative analysis of protein expression including GPX4, podocin, and nephrin. **P < 0.01.

## Discussion

DN is a common chronic complication of diabetes mellitus [35]. Mitochondrial injury-induced podocyte apoptosis is considered the most destructive factor in DN progression [36]. In this study, we found that germacrone could mitigate the symptoms of STZ-induced type Ι DN. The protective effect of germacrone was correlated with mitochondrial injury repair in podocytes. In addition, miR-188-3p negatively regulated germacrone-mediated resistance to mitochondrial damage and apoptosis in podocytes. This study indicates that germacrone may serve as an anti-apoptotic drug targeting podocytes for DN therapy.

Germacrone, a herbal volatile oil, is a constituent of massive aromatic compounds purified from the rhizomes of Curcuma zedoaria oil (C. oil) [19,37]. It has been reported that germacrone can inhibit p-glycoprotein expression or mediate pro-apoptotic protein expression to repress cancer cell proliferation [38–40]. Germacrone can reinforce the expression of anti-inflammatory mediators and suppress pro-inflammatory cytokine levels to exert anti-inflammatory effects [41,42]. Renal inflammation-induced podocyte apoptosis and loss contribute to the development of DN [43]. In this study, germacrone treatment relieved DN symptoms, restored the glomerulus morphological structure, and inhibited HG-induced podocyte apoptosis, which implied that germacrone might play a protective role in podocytes of type I DN. It is possible that the protective mechanism is related to the anti-inflammatory action of germacrone.

Pro-inflammatory cytokines play a pivotal role in the generation of reactive oxygen and nitrogen species, and oxidative damage subsequently causes mitochondrial DNA integrity and mitochondrial dysfunction [44]. Germacrone possesses consequential antioxidant actions in transient focal ischemia in the rat brain [45]. It is possible that germacrone-mediated antioxidant capability has repair effects on mitochondrial injury. Here, we found that germacrone could repair mitochondrial damage and strengthen antioxidant capacity to inhibit the production of oxidation products, thereby preventing podocyte apoptosis and relieving DN. This is in agreement with previous observations. Therefore, we speculated that the antioxidant effect of germacrone ameliorated mitochondrial injury in podocytes and, subsequently, the progression of type I DN.

There are substantial data supporting the profound role of podocytes in the foremost mechanisms in DN [9]. Hypertrophy, epithelial-mesenchymal transition, detachment, and loss of podocytes are involved in the pathomechanism of DN [46–48]. Recently, increasing attention has been focused on the relationship between ncRNAs, chronic nephritis, and diabetic glomerular injury. miRNAs, which are the predominant ncRNAs, can bind to target mRNAs, inhibit their expression, and participate in the progression of DN [49,50]. miR-188-3p plays an anti-apoptotic role in numerous cell types [51]. Knockdown of taurine upregulated gene 1 inhibits proliferation and facilitates apoptosis through the miR-188-3p/FGF5 pathway in islet cells of type II diabetes mellitus [52]. miR-188-3p is implicated in the progression of diabetes mellitus, however, its role in DN remains unclear. In the present study, miRNA-188-3p was upregulated in STZ-induced type Ι DN mice. Germacrone-mediated protective progression in DN was implicated in the miRNA-188-3p downregulation, indicating that miRNA-188-3p might mediate the improvement of DN afforded by germacrone. A considerable number of studies have revealed that mitochondrial injury has emerged as a high-priority factor in the pathogenesis of podocytes in DN [53]. Additionally, miRNA-188-3p agomir also abolished the germacrone-mediated repair of mitochondrial injury. It is possible that miRNA-188-3p upregulation induced mitochondrial injury, resulting in podocyte apoptosis in type I DN mice. The combination of miR-188-3p antagomir may have a synergistic effect with germacrone in treating type I DN.

Excessive ROS leads to a decrease in GPX4, which is an important antioxidant, and GPX4 reduction causes mitochondrial damage [54]. Mice exhibited renal failure due to the absence of GPX4. Mitochondrial dysfunction further hinders the synthesis of GSH, a substrate of GPX4, which in turn triggers ferroptosis and the accumulation of membrane lipid ROS [55,56]. Ferroptosis is a new form of cell death triggered by iron-dependent lipid peroxidation [57]. Here, germacrone induced an increase in GPX4 in type I DN mice, and miR-188-3p overexpression neutralized the upregulation of GPX4 mediated by germacrone. It is possible that GPX4 alteration-mediated ferroptosis may regulate the treatment process of germacrone or miR-188-3p antagomir in type I DN. However, our research did not address certain key issues. First, we did not directly elucidate the origin of cells with mitochondrial damage in the mouse model. Second, the living inflammatory microenvironment may cause damage to podocytes. Other cell types, such as glomerular interstitial cells or glomerular endothelial cells, could also release pro-apoptotic factors that cause a loss in podocytes. Third, we did not determine whether the overexpressed miR-188-3p in STZ-induced DN mice was specifically located in podocytes. It is possible that increased miR-188-3p may be widely expressed in the glomerulus. In addition, the fundamental mechanism was not thoroughly explained, and the downstream target genes of miR-188-3p require in-depth investigation. Therefore, whether germacrone adjusts mitochondrial function through miRNA-188-3p to protect podocytes and ameliorate DN remains to be further explored.

## Conclusion

In summary, the current study revealed that germacrone protects against mitochondrial malfunction and podocyte apoptosis in type I DN. Mechanistically, miR-188-3p dramatically abolished the effects of germacrone, triggering oxidative stress and eventually podocyte apoptosis. Our findings may provide innovative ideas for the treatment of DN in type I diabetes.

## Supplementary Material

Supplemental Material

## Data Availability

All data generated or analyzed during this study are included in this published article and its additional files.
